# Visualization Method of Key Knowledge Points of Nursing Teaching Management System Based on SOM Algorithm and Biomedical Diagnosis

This article has been retracted.

**DOI:** 10.1155/2022/7057437

**Published:** 2022-10-11

**Authors:** Die Hu, Le Fang

**Affiliations:** ^1^Department of Nursing, Zhengzhou Health Vocational College, Zhengzhou 450122, China; ^2^Ophthalmology Department, People´s Hospital of Zhengzhou, Zhengzhou 450122, China

## Abstract

The traditional nursing teaching knowledge point recommendation algorithm based on collaborative filtering is difficult to deal with the problem of data sparsity, while the traditional recommendation algorithm based on matrix decomposition has poor scalability in dealing with high-dimensional data, and their recommendation results are only determined according to the prediction score, resulting in low recommendation accuracy. In view of this, a nursing teaching knowledge point recommendation method based on a SOM neural network and ranking factor decomposition machine is proposed. Firstly, the SOM neural network is used to cluster users based on users' academic background information, then the partial order relationship of nursing teaching knowledge points is constructed by using users' explicit and implicit web access behavior, and finally, the factor decomposition machine is used as the ranking function to classify users' academic background web access behavior, borrowing nursing teaching introduction text, and other characteristic information were modeled, and the peer-to-peer ranking learning algorithm was used to accurately recommend nursing teaching knowledge points. Experimental results show that the proposed method can effectively alleviate the problem of data sparsity and improve the accuracy and efficiency of recommendations.

## 1. Introduction

With the continuous advancement of the digital construction of nursing teaching knowledge points, the number of electronic nursing teaching knowledge points has increased sharply, resulting in problems such as information overload and cognitive loss when users search for nursing teaching knowledge points [1]. Therefore, how to provide users with nursing teaching knowledge point recommendation services according to the users' preferences for nursing teaching knowledge points has become an important problem to be solved to improve the personalized service quality of nursing teaching knowledge points. Most of the existing personalized nursing teaching knowledge point recommendations are realized by the traditional recommendation method based on user collaborative filtering. The basic principle is to find the nearest neighbor users similar to the target users by calculating the similarity between users, then predict the score value of the target users on the nursing teaching knowledge points according to the historical score data of the similar users on the nursing teaching knowledge points, and recommend the nursing teaching knowledge points based on the score value. Because in the case of sparse data, a user-based collaborative filtering algorithm [2]. Therefore, most scholars are committed to improving the above algorithms. For example, song Chuping integrates reader characteristics and nursing teaching characteristics into user similarity calculation to improve the accuracy of recommendation [3]. However, with an increase in the number of users, the amount of user similarity calculation will increase , resulting in a reduction in recommendation efficiency. Therefore, the SOM algorithm is used for clustering. By calculating the similarity between the target user and each clustering center, the cluster is found, and the nearest neighbor user set is constructed, so as to reduce the amount of user similarity calculation. However, because the traditional algorithm is affected by the initialization K value and the clustering time is long, the accuracy of clustering results is not high [4].

## 2. Visualization of Key Knowledge Points of Nursing Teaching Management System

### 2.1. SOM Structure of Key Knowledge Points of Nursing Teaching Management System

A nursing knowledge map is a specific knowledge base for the nursing field, which includes a series of entities in the nursing field and their associations. There is a precedent for the construction of a nursing knowledge map [5]. Using the technologies of text extraction, relational data conversion, and data fusion, this paper explores the automatic construction method and standardized process of a TCM knowledge map in order to realize the template-based TCM knowledge Q&A and the auxiliary prescription based on the knowledge map reasoning [6]. The SOM network structure is shown in Figure 1.

A SOM network is a tissue feature mapping network. Its basic principle is that for each input vector, a neuron in the output layer has the closest value to the input vector and wins by receiving the maximum stimulation. Some neurons around the winning neuron are also greatly stimulated due to lateral action. At this time, the network performs a learning operation, and the winning neuron and its surrounding neurons modify their own weight vector to move to the input vector [7]. Each neuron is moved to the whole input space as more vectors are submitted, and it is close to the input vector of its nearest vector value and arranged in that layer to obtain a classification. According to experience, when all input and output values are between 0 and 1, the calculation effect of the SOM neural network is the best [8]. Assign the weights of each neuron in the network to the random number in the [0,1] interval as the initial value *w*_*ij*_, set a large neighborhood radius *n*, and set the number of neurons that are learning *t*. Randomly select a training mode *x*(*t*) = (*x*_1_(*t*), *x*_2_(*t*),…, *x*_*n*_(*t*)) to provide to the input layer of the network. Select the neuron matching the input vector as the winning neuron *c*. If the Euclidean distance is adopted, *C* is

(1) $$\begin{array}{c} \left\|x\left(t\right)-w_{c}\left(t\right)\right\|=\min\;\left\{\left\|x\left(t\right)-w_{j}\left(t\right)\right\|\right\}. \end{array}$$

Update the weights of neurons in the neighborhood to make them move in the direction of super input vector. Assuming that an n-dimensional input eigenvector can be expressed as *x* = (*x*_1_,*x*_2_,…,*x*_n_)∈*R*_*n*_, *y*_i_ as the target prediction value corresponding to the input eigenvector, FM can use the decomposition interaction parameters to model all nested interactions of *n* input variables of *x* in d-dimension [9]. When *d* = 2, the factorization machine model can be expressed as follows:

(2) $$\begin{array}{c} \hat{y}\left(x\right)≔w_{0}+\overset{n}{\underset{i=1}{\sum }}w_{i}x_{i}+\overset{n}{\underset{i=1}{\sum }}\overset{n}{\underset{j=i+1}{\sum }}w_{i,j}x_{i}x_{j}. \end{array}$$

Where *w*_0_ is the total deviation; *w*_*i*_ is the unary interaction parameter of the input variable *x*_i_; *w*_*ij*_ is the decomposition parameter between *V*_*I*_ and *V*_*J*_, which is defined as follows:

(3) $$\begin{array}{c} w_{i,j}=<v_{in}v_{j}>=\overset{k}{\underset{f=1}{\sum }}v_{i,f}\cdot v_{j,f}. \end{array}$$

Where *k* is a super parameter that defines the decomposition dimension. Suppose there is an input space X ∈ *R*_N_, where *n* is the number of features. At the same time, there is an output space (i.e. scoring space) in which the tag *Y* = {*r*_1_,*r*_2_,…,*r*_q_} represents the user's preference order for items, and the fixed order they maintain is *r*_q_,r_q−1_,…,*r*_1_ where *v* represents the preference relationship. In order to determine the order relationship between items, we need to select a set of sorting functions f ∈ F so that each candidate function *f* in *f* can determine the following partial order relationship, namely:

(4) $$\begin{array}{c} x^{\left(i\right)}>x^{\left(j\right)}⟺f\left(x^{\left(i\right)}\right)>f\left(x^{\left(j\right)}\right). \end{array}$$

Suppose, in *x*× there is a set of sorting reals *S* = {(*x*(*i*), *y*(*i*))}, *T*_i_ = 1 in *y* space, where *y*(*i*) is the preference sorting, and *t* is the number of instances. The sorting task is to find an optimal function f*∗* ∈ f to minimize the loss function of a given sorting instance. Here, *F*_m_ function is selected as the sorting function, which is as follows:

(5) $$\begin{array}{c} f_{\theta }\left(x\right)≔w_{0}+\overset{n}{\underset{i=1}{\sum }}w_{i}x_{i}+\overset{n}{\underset{i=1}{\sum }}\overset{n}{\underset{ji+1}{\sum }}x_{i}x_{j}\overset{k}{\underset{f=1}{\sum }}v_{I,f}v_{j,f}. \end{array}$$

Convert any instance pair and their sequential relationship into a new instance, and give the instance a new label. Assuming that *p* and *q,* respectively, represent an instance in an instance pair, and *y*_p_ and *y*_q_ represent their sorting, there are

(6) $$\begin{array}{c} \left(p,q\right),z=\left\{\begin{array}{cc} +1 & y_{p}>y_{q},\\ -1 & y_{\phi }>y_{j}. \end{array}\right. \end{array}$$

According to the above method, a new training set s' = {*P*(*t*), *q*(*t*), and *Z*(*t*)}, *L*_i_ = 1, can be created from a given training set *s*, where *l* is the number of newly constructed instances. Thus, the hinge loss function of the t-th instance pair in the training set s' is

(7) $$\begin{array}{c} l_{i}\left(f;p^{\left(1\right)},q^{\left(0\right)},z\right)={\left[1-z\times \left(f_{\Theta }\left(p^{\left(\omega \right)}\right)-f_{\Theta }\left(q^{\left(\theta \right.}\right)\right)\right]}_{+}. \end{array}$$

Where the subscript “+” represents the positive part; f(P(t)) - f(q(t)) can be calculated by FM function within the linear time complexity *O* (*k*•*n*). Define a global loss function on the whole training set s':

(8) $$\begin{array}{c} \min_{\Theta }\;L\left(\Theta \right)=\overset{l}{\underset{i=1}{\sum }}l_{r}\left(f;p^{\left(t\right)},q^{\left(\theta \right)},z^{\left(b\right)}\right)+\underset{\theta \in \Theta }{\sum }\lambda_{\phi }\theta^{2}. \end{array}$$

Where *λ*,*θ* re model parameters, *θ* regularization parameters, and initial parameters, knowledge point feature extraction based on the above algorithm can better comb and display the context.

### 2.2. Characteristic Identification of Knowledge Points in Personalized Nursing Teaching

The purpose of personalized nursing teaching knowledge point recommendation based on the SOM neural network and ranking factor decomposition machine model is to accurately cluster users by using the nonparametric characteristics and high accuracy of the SOM neural network, and then use the characteristics of the factor decomposition machine that can easily integrate high-dimensional data as a ranking function to evaluate the academic background, quality, and accuracy of users in the same cluster. Borrow a variety of characteristic information, such as nursing teaching introduction text and web access behavior to model, and use the level sorting learning algorithm to train the model so as to realize the accurate sorting and recommendation of nursing teaching knowledge points. The flow chart of sorting recommendations based on SOM and RFM is shown in Figure 2.

**Step 1 .**

initialize the network, that is, set the SOM network and initialize the initial value of each training parameter [10, 11]. The values to be initialized are: the random number that gives the link weight W in the [0,1] interval; determine the initial value of the learning rate *n* (1)*η* (o) (0 < *η* (*ω*)< 1); and determine the initial value *n* (*o*) of the domain *n* (*t*), where *G* is the winning neuron; calculate the Euclid distance between the weight vector *w* = (*w*, *m*) and the input sample *x* = (*x*_1_, *x*_2_,…, *x*_*n*_), and select the minimum distance to determine the winning neuron [12]. Adjust the connection weight *w* and update the neighborhood *n* (*i*) of the output layer. The update formula for the connection weight between each neuron in the input layer and the neuron in the input layer is as follows:

(9) $$\begin{array}{c} \left\{\begin{array}{c} w_{ij}\left(t+1\right)=w_{ij}\left(t\right)+\eta \left(t\right)\times \left(x_{j}-w_{ij}\left(t\right)\right)\text{,}\\ gw_{ij}\left(t+1\right)=w_{ij}\left(T\right)+\eta \left(t\right)/2\times \left(x_{j}-w_{ij}\left(t\right)\right),j\in N_{g}\left(t\right),\\ w_{ij}\left(t+1\right)=w_{ij}\left(t\right),j\notin N_{g}\left(t\right). \end{array}\right. \end{array}$$

Where *w*_*ij*_(*t*+1) represents the input neuron at *t* + 1 time; connection weight with output neuron *J*; *n* (*t*) is the domain range centered on the winning neuron *g* at time *t*; update the learning rate *M* and domain *n* (*t*); then,

(10) $$\begin{array}{c} \left\{\begin{array}{c} \eta \left(t\right)=\eta \left(0\right)\times \left(1-t/T\right),\\ N_{g}\left(t\right)=N_{g}\left(0\right)\times \left(1-t/T\right). \end{array}\right. \end{array}$$

The knowledge points have an inevitable sequence in the learning process. Whether a knowledge point can be learned at present often depends on whether other knowledge points have been learned, or if the latter is the preparatory knowledge of the former [13]. Before learning a certain knowledge point, you must first learn another related knowledge point, and the relationship between the two is the precursor relationship [13]. After learning a certain knowledge point, the knowledge points directly supported by this knowledge point form a successor relationship between the two, as shown in Figure 3.

As a knowledge system, there is an inherent relationship of mutual restriction and mutual influence between concepts and principles [14–16]. The relationship reveals that there is a network structure between knowledge points and points out that knowledge is composed of a group of interconnected and interactive nodes. A correlation is conducive to the mastery of knowledge and the formation of knowledge system. The association relationship between knowledge points can be divided into two categories: one-to-one association (1 : 1), which means that one knowledge point only corresponds to another knowledge point; one to many association (1 : m), which indicates that a knowledge point can be associated with multiple knowledge points; and the graph indicates the one to many association between knowledge points.  Figure 4 shows the characteristics of the tree structure of nursing knowledge points.

Knowledge points are very important for teaching activities. After completing the division of knowledge points and determining the relationship between knowledge points, we should consider how to organize teaching according to knowledge points in a specific knowledge field, because teaching is composed of the teaching of knowledge points [17–19]. The knowledge point structure model can better organize and describe the content of knowledge fields. The knowledge point structure model is basically a hierarchical tree structure. In the hierarchy of relationship, the parent-child relationship and the brother relationship are the two most important relationships. They serve as the basis for building the tree structure for knowledge points. The association relationship enriches the content of the knowledge tree. Using these two relationships to describe knowledge points constitutes a knowledge point structure model. On the basis of this model, the knowledge points of a specific discipline can be listed and organized according to the relationships between knowledge points, and the knowledge point structure diagram of this discipline can be constructed. The knowledge in textbooks is generally arranged in linear order. In fact, the relationship between knowledge points is complex [20, 21]. To learn a knowledge point, you must first have certain basic knowledge (a precursor relationship), that is, master some knowledge points. To learn these knowledge points, you may need to master other knowledge points. In this way, all knowledge points and the relationship between them constitute a knowledge point network. The knowledge point network is a network composed of several related knowledge points based on their internal relations [19]. The nodes of the network represent knowledge points, and the links between nodes represent the links between knowledge points. After learning a knowledge point, students should also understand that the “environment” of the knowledge point is the content of its sequence, left and right, up and down, so as to determine the mark of the “status” of the knowledge, in order to make students realize the structure of the same network between the knowledge points and establish the consciousness of the network. Through this network diagram, teachers and students can have a clear understanding of some theorems of solid geometry [22, 23]. For example, in the teaching process, if we pay attention to the application of the knowledge point network to tell students about knowledge points, it is beneficial for students to understand the knowledge structure, build their' own cognitive systems, and facilitate the transfer of memory and knowledge skills, because the knowledge point network contains information about the learning path , and this learning path should be reasonable and optimal for students. In a word, this paper deeply analyzes the relevant contents of knowledge point representation and establishes a knowledge point model that is suitable for teaching in form, reflects the connotation of knowledge points in content, and helps to realize the teaching process, which provides a new perspective for teachers to design teaching according to the attributes and laws of knowledge points.

### 2.3. Realization of Knowledge Point Context Visualization

The construction of a knowledge map is generally divided into two ways: top-down and bottom-up. The top-down construction method is based on ontology and takes highly structured encyclopedias and other websites as data sources to extract ontology and rule constraints and fill them into the knowledge base.

Figure 5 shows the technical architecture of the knowledge map. The three steps of knowledge extraction, fusion, and processing in the box are the core of the construction of the knowledge map. It can be seen from the figure that structured data can easily extract knowledge from it because of its high degree of standardization; semistructured and unstructured data have poor standardization and are difficult to obtain knowledge directly. Therefore, it is necessary to extract the entities and associations of knowledge with the help of a series of operations such as attribute extraction, relationship extraction, and entity extraction, and then store them in the knowledge base. The construction process of a knowledge map is a continuous cycle. The iterative process can be roughly divided into three stages: knowledge extraction, knowledge fusion, and knowledge processing.

In the traditional teaching of nursing management, the teaching goal is above all else. It is not only the starting point of the teaching process but also the destination of the teaching process. However, in the classroom of network teaching, because it emphasizes that students are cognitive subjects and active constructors of meaning, students' meaning construction of knowledge is regarded as the ultimate goal of the whole learning process. The whole teaching process starts with a situation conducive to students' meaning construction and closely surrounds the center of “meaning construction.” Whether it is students' independent exploration, cooperative learning, or teachers' guidance, in short, all aspects of the learning process should belong to this center, which should be conducive to completing and deepening the meaning construction of the learned knowledge. Combined with the characteristics of nursing management and based on constructivism theory, this paper constructs the structure of nursing management teaching modes in a network environment. The specific operation flow is shown in Figure 6.

Acquiring knowledge through a well-structured relational database or third-party knowledge base is also a good choice to build a knowledge map.

Merge the ontology in the third-party knowledge base into its own library. As another important knowledge source for knowledge mapping, relational databases can usually use the resource description framework (RDF) as a data model and integrate it into a knowledge map. At present, a considerable number of open-source tools support the transformation of data in structured relational databases into RDF triples to realize the construction of a knowledge map. This view is a local view, which is only used to show the association between the outcome entity and the interaction entity in a specific domain. In the above view, it can be seen that for a certain nursing symptom, the associated nursing measures are very concentrated in some fields, and the visual recommendation of nursing measures can be made for the nursing measures in the same field. Therefore, we hope to design a view that can not only provide a more detailed expression of information, but also reflect the hierarchical information of nursing measures and their fields. The package layout view has the ability for hierarchical expression and can classify and display data according to categories. However, the package view is not suitable for expressing network class information. Atlas data is a kind of network data. Network data can be expressed by force guidance diagrams, radar diagrams, chord diagrams, etc. Among them, the force guidance diagram is a node connection diagram, and the package diagram is a content filling diagram. If the two are used as a mixed view, they can achieve a complementary effect visually. Therefore, consider combining the two views. At the view level, the system interface is mainly divided into three parts. On the right is a general introduction to the Atlas data, which is divided into the data source, data description, overall data analysis, and node selection details. The lower side is the system toolbar, which switches the interaction mode of the system. The middle part is the data view, which is used for data display and data view interaction.

## 3. Analysis of Experimental Results

In order to verify the effectiveness of the proposed SOM method, comparative experiments are carried out. FM is a traditional factorization machine model, which is used to judge that SOM based on ranking learning has higher accuracy than traditional FM; BPRMF is a matrix decomposition model based on pairwise ranking method, which is used to judge the influence of ranking learning algorithms on recommendation accuracy; and RSVM is a support vector machine based on pairwise ranking method, which is used to judge that FM, as a ranking function, can more accurately express user preferences than SVM, as shown in Table 1.

For ranking recommendation, because users pay more attention to the recommendation quality of the top-ranked items in the recommendation list, this study selects two ranking position-sensitive evaluation indicators for evaluation, namely average accuracy and normalized impairment cumulative gain. Map is defined as follows:

(11) $$\begin{array}{c} MAP=\frac{\overset{N}{\underset{r}{\sum }}\left(N_{r}/r\times l\left(r\right)\right)}{N_{a}}. \end{array}$$

Where *r* is the sorting ordinal number; *N* is the number of recommended products; NR is the number of related commodities sorted as *r*; *n*_r_/*r* is the accuracy of truncated sorting; *l* (*r*) is a binary correlation function with a sorting number *r*; correlation is 1 and uncorrelation is 0; Na is the total number of related commodities. The larger the map value, the higher the ranking of items related to user preferences, and the better the overall ranking effect of the algorithm. *N*_dcg_ is defined as follows:

(12) $$\begin{array}{c} NDCG@P=\frac{1}{Z_{P}}\overset{p}{\underset{i=1}{\sum }}\frac{2^{k\left(i\right)}-1}{lg\left(1+i\right)}. \end{array}$$

Where P represents the position of the item in the list, *Z*_*p*_ is the normalization factor, and *K* (*i*) represents the correlation level between the item with location *i* and user preference. The value range of NDCG is [0,1]. The larger the value, the more consistent the sorting results are with the user's interests and preferences. Their entity information comes from the nursing guide. By grasping the nursing guide, we extract different sets of nursing entities and the contact edge sets between entities and construct the entity network in the nursing field. The extracted main entity information and the association information between some entities are shown in Table 2.

The traditional algorithm cannot be directly applied to the research object of this paper. In order to verify the effectiveness of the improved algorithm, this section will compare the clustering quality of the improved k-medoids algorithm with that of the improved SOM algorithm. The interclass distance and intraclass distance of the SOM improved algorithm and the k-medoids algorithm are shown in the following Table 3. In the experiment, the two algorithms are clustered ten times, and the average values of SSE and SSB from multiple experiments are calculated. As shown in Table 4, the experimental results of the two algorithms are compared.

From the perspective of stability, the repetition rates in the clustering results of the SOM improved algorithm and the *k*-medoids improved algorithm are compared. Here, eleven experiments are also carried out on different algorithms to calculate the average repetition rate of different algorithms.

In many experiments and simulations, the clustering results of the SOM improved algorithm can obtain a 67.0% repetition rate, which is similar to the clustering effect of the *k*-medoids improved algorithm, which proves that the SOM improved algorithm in this paper also has good stability. The following figure shows the proposed SOM algorithm and the comparison algorithm MAP@10 and NDCG@10 results on evaluation indicators.

It can be seen from Figure 7 that the performance of the algorithm varies with the value of *K*. When *k* = 15, the performance of the four algorithms is the best. At the same time, it can be seen that SOM obtains the best performance under different *K* values. This is because, compared with FM, SOM adopts a pairwise sorting learning algorithm, so its performance is better than FM; compared with BPRMF, SOM can not only integrate the explicit and implicit feedback information of users but also integrate the text information of the borrowing nursing teaching introduction and the borrowing log information, so its performance is also better than the traditional methods. At the same time, SOM's sorting function FM uses interaction parameters rather than independent parameters to model the interaction between features, so SOM can obtain better performance. Especially in the case of sparse data, its performance is better.

## 4. Conclusion

In the courses that need a lot of practice, the implementation of a project-based teaching method can quickly improve students' practical operation abilities. At the same time, the establishment of students' theoretical knowledge systems cannot be ignored. The nursing specialty is a highly practical specialty. It adheres to the project-based teaching method without making students with weak theoretical basic knowledge more backward. Cultivating practical talents is one of the ways to realize this. The cultivation of operation skills is an important task in nursing teaching. Students' nursing operation level directly affects the effects of clinical practice and the future development of nursing specialties, as well as the quality of their practical talents. Years of nursing practice show that nursing teaching management is a systematic, phased, complex, and carefully organized process. In order to ensure the effect of nursing operation teaching, this paper uses a SOM neural network to cluster users according to the users' academic background information, analyzes the explicit and implicit web access behavior of nursing teaching knowledge points, constructs the partial order relationship of nursing teaching knowledge points, classifies users' academic background web access behavior, and uses a point-to-point sorting learning algorithm to accurately recommend nursing teaching knowledge points. Different teaching purposes can be implemented for each type of students. Students with weak theoretical knowledge can purposefully integrate, so that excellent students can help weak students learn from each other, effectively improve the project teaching level, help students, promote students' healthy growth, and learn professional nursing skills.

## Figures and Tables

**Figure 1:** The SOM network structure.

**Figure 2:** Accurate recommendation process of teaching resources based on SOM.

**Figure 3:** Leading and following relationships between knowledge points.

**Figure 4:** Tree structure characteristics of nursing knowledge points.

**Figure 5:** Structure diagram of a knowledge map visualization technology.

**Figure 6:** Basic flow chart of nursing teaching view processing under the SOM network environment.

**Figure 7:** Comparison of knowledge point context view and useable effect.

**Table 1:** System test environment.

name	To configure
Processor	Intel(R)Core(TM) i7-7700HQ
Hard disk	1024 GB
Memory	32G
Operating system	Windows 7
Web server	Flask
Database	MySQL

**Table 2:** Data information of nursing entities.

Number of entities in nursing symptom area	Number of nursing symptom entities	Number of nursing measures symptom entities	Number of nursing measures entities	Number of symptom domain associations	Number of symptoms associated with measures
8	130	8	410	128	2226

**Table 3:** Comparison of effectiveness between the SOM improved algorithm and the k-medoids improved algorithm.

	SSE	SSB
SOM improved algorithm	9102	13024
Improved k-medoids algorithm	9325	12058

**Table 4:** Comparison of stability between the improved algorithm of the SOM and the improved algorithm of k-medoids.

	Repetition rate (%)
SOM improved algorithm	67.0
Improved k-medoids algorithm	66.6

## Data Availability

The data used to support the findings of this study are included within the article.
